# Big Data, Extracting Insights, Comprehension, and Analytics in Cardiology: An Overview

**DOI:** 10.1155/2021/6635463

**Published:** 2021-01-30

**Authors:** Hui Xiao, Sikandar Ali, Zhen Zhang, Muhammad Shahzad Sarfraz, Fang Zhang, Mohammad Faisal

**Affiliations:** ^1^Zhongnan Hospital of Wuhan University, Information Center, Wuhan 430071, China; ^2^Department of Computer Science and Technology, China University of Petroleum-Beijing, Beijing 102249, China; ^3^Department of Computer Science, National University of Computer and Emerging Sciences Islamabad, Chiniot-Faisalabad Campus, Chiniot, Pakistan; ^4^Department of Computer Science and Information Technology, University of Malakand, Chakdara, Pakistan

## Abstract

Healthcare system facilitates the treatment of patients with the support of wearable, smart, and handheld devices, as well as many other devices. These devices are producing a huge bulk of data that need to be moulded for extracting meaningful insights from them for the useful use of researchers and practitioners. Various approaches, methods, and tools are in use for doing so and to extract meaningful information in the field of healthcare. This information is being used as evidence to further analyze the data for the early care of patient and to devise treatment. Early care and treatment can facilitate healthcare and the treatment of the patient and can have immense potentiality of dropping the care cost and quality refining of care and can decrease waste and chances of error. To facilitate healthcare in general and cardiology in specific, the proposed study presents an overview of the available literature associated with big data, its insights, and analytics. The presented report will help practitioners and researchers to devise new solutions for early care in healthcare and in cardiology.

## 1. Introduction

The increase in use of smart devices such as sensor, actuator, and wearable devices, as well as other devices, has produced massive amount of data that need to be shaped in a structure way to mine the information and useful insights for the useful use of research and practice. This increase of information can yield research issues and challenges as extracting useful information becomes a challenging task for research. The useful insights once drawn in a successful way can ultimately care the patient and provide effective treatment in the early stage. Diverse approaches, methods, and mechanisms are in practice to tackle the issues of big data and its analytics in the field of healthcare in general and cardiology in specific.

The role of data processing and information in healthcare has always been vital in healthcare for decision-making and its provision. Medical big data is produced from the communication and digitization in healthcare. Healthcare providers and hospital industry provide a huge amount of data from other segments, such as medical equipment, medical insurance medical research, and life science. Huge amount of data exists, which grasps the potential of support of healthcare and medical tasks. The integration of machine learning, artificial intelligence, and advanced analytics offers numerous opportunities for transmuting such data into actionable and expressive insights for supporting decision-making. This can ultimately make availability of patient care at high quality and real-time situation response and can protect lives on the clinical side and develop the services and processes, improve the use of resources, and minimize the costs on the maintenance and financial front [1, 2].

With the rise of advanced approaches such as analytical techniques and approaches, the stakeholders of healthcare can not only connect the data power for historical analysis of data but also predict future outcomes with predictive analytics for defining best accomplishment for present situation [3, 4]. Conventionally, the practitioners of clinic rely on reserved information accessible to them and their past involvement for treatment of patients. Data availability from diverse sources deals with the chance to have a complete thought of patient well-being. The use of cutting-edge technologies against such data aids access to the appropriate information at precise place and accurate time for delivering precise care [5].

The proposed study presents an overview of the available literature associated with big data, its insights, and analytics. The process of search for the proposed study was done in the popular libraries with the aim of obtaining associated materials. The presented report will help practitioners and researchers to devise new solutions for early care in healthcare and in cardiology.

The remainder of the paper is organized as follows: Section 2 presents the interrelated research to current study.  Section 3 presents library-based search process for the proposed study.  Section 4 concludes the paper.

## 2. Related Work

Several approaches have been in practice to tackle diverse issues of big data and its analytics in healthcare. Pevnick et al. [6] offered a review that discusses the current and upcoming devices intended for measuring the actions of heart rhythm, heart rate, and thoracic fluid. Various frameworks were presented, which classify and understand the wearable devices. Mehta et al. [7] presented a systematic mapping study for analyzing and identifying the research studies on analytics of big data and use of artificial intelligence in healthcare. The study identified 2421 papers for the year's ranges from 2013 to February 2019. These papers were evaluated, and the results show that the study will support the necessity in the use of technologies in healthcare. Atitallah et al. [8] surveyed the literature associated with the DL and IoT applications for smart cities' developments. Initially, the basics of IoT were defined followed by the characteristics of IoT-produced big data. After that, the various structures used for analytics of IoT big data were presented. The common DL models were surveyed and reviewed the current research employing the IoT and DL for developing services and smart applications for smart cities. The existing issues and challenges encountered throughout the smart city's development were outlined. Kazmierska [9] presented a study on the needs of community in translating multisource data into clinical decision aids.

Ben-Assuli et al. [10] demonstrated power prediction of four popular algorithms and matched their accuracy in congestive heart failure predicting initial patient mortality. The results show that the current models outperform those described in the literature. The results further support the policy-makers in allocation of resources for establishment of comprehensive systems of integrated health IT aiming at simplification of analytics of ML. Dipti Itchhaporia [11] analyzed the existing application and state of machine learning approaches and artificial intelligence in cardiovascular medicine. The effects of emerging technologies on cardiovascular medicine are emphasized for providing understanding to the clinical practice and to find probable patient assistances. Nazir et al. [12] provided a wide-ranging overview of the available big data studies in cardiology. The study followed a protocol of systematic literature review for presenting the published material from 2008 till 2018 associated with big data features, applications, and analytics in cardiology field. The authors identified 190 potential studies and analyzed them. These studies were published in conferences, books, journals, and many other online materials. The study was presented as an evidence for the researchers and practitioners to devise novel solutions in the area of interest. Nazir et al. [13] presented a comprehensive review of the 10 years from 2008 to 2018 associated with the visualization of big data in the area of cardiology. The study identified 53 prospective papers related to visualization of big data in cardiology. The study was based on protocol with defined research questions, inclusion and exclusion criteria, and quality criteria. These identified studies were analyzed according to the defined research questions. The study highlighted the increase of the number of researches in the area and focused on further research and innovations in the field. These studies were done in order to support the usage of big data in healthcare.

Bizopoulos and Koutsouris [14] surveyed applications of deep learning that uses structured data and signal and imaging modalities from cardiology. The benefits and limitations of applications of deep learning in cardiology and in medicine in general are discussed. Cannière [15] examined the developments of heart rate variability factors during short-term interval all the way through cardiac rehabilitation. Electrocardiography signals, documented with the help of wearable device in 129 patients following cardiac rehabilitation program, were analyzed. The findings of the study present appreciated insights into disease monitoring during cardiac rehabilitation in future application.

## 3. Library-Based Search Process

This study offers to present an overview of the existing approaches and methods for big data, its analytics, and insights in cardiology. Various popular libraries such as ScienceDirect, IEEE, Springer, and Wiley were searched with the aim of obtaining associated materials interconnected to the current study. The information gathered from these libraries was analyzed and presented from different perspectives in the form of different tables and figures. This information includes the type of article, number of publications, topics covered, subject areas, and publication titles. Initially, the library of ScienceDirect was checked and the following information was obtained.  Figure 1 depicts the types of articles with publications. The figure shows that a bigger number of publications were in the form of research article.

Figure 2 presents the articles in total with the given year. More publications are shown in the year 2020, which shows the increase in number of researches.

Figure 3 depicts the subject areas with the number of publications.

The library of IEEE was searched for the purpose of identifying relevant information.  Figure 4 represents the information of publication topics with the total number of articles published.

The paper type and total number of publications in the same library are shown in Figure 5.

Figure 6 presents the conference location with the number of publications.

After this, the library of Springer was searched to view the information for the purpose of analysis.  Figure 7 depicts the type of articles with the number of publications.

The discipline with the total number of articles is shown in Figure 8. The purpose of this search was to identify the disciplines covered by the area.

The libraries of Wiley and Taylor & Francis were also part of the proposed study. These libraries were searched for relevant information and analysis.  Figure 9 depicts the publication types with total number of articles published. In the figure, it is shown that more papers are published with type journal.

Figure 10 presents the number of publications in the given years from 2016 till 2020.

After the statistics were obtained, the papers were reviewed and the details with short descriptions of the papers were given.  Table 1 shows the big data and its analytics in cardiology.

Big data are considered to be the main asset of the organization for its successful operations and future endeavour [72–77].

## 4. Conclusion

Healthcare system facilitates the patients with the support of wearable devices, smart devices, handheld devices, and many other devices. These devices are producing a huge bulk of data that need to be moulded for extracting expressive insights from them for the useful use of researchers and practitioners. Various approaches, methods, and tools are in use for doing so and to extract meaningful information in the field of healthcare. This information is being used as evidence to further analyze the data for the early care of patients and to devise treatment. Early care and treatment can facilitate healthcare and patient and can have immense potentiality of quality refining of care and lessen care cost and can decrease waste and chances of error. To facilitate healthcare in general and cardiology in specific, the proposed study presents an overview of the existing literature associated with big data, its insights, and analytics. The presented report will help practitioners and researchers to devise new solutions for early care in healthcare and in cardiology.

## Figures and Tables

**Figure 1:** Article types.

**Figure 2:** Number of papers published.

**Figure 3:** Subject area with number of articles.

**Figure 4:** Publication topic with number of articles.

**Figure 5:** Paper type with number.

**Figure 6:** Conference location with number of articles.

**Figure 7:** Content type.

**Figure 8:** Discipline with number of articles.

**Figure 9:** Publication type with number of papers.

**Figure 10:** Publication in the year.

**Table 1:** Work in the area of big data and its analytics in cardiology.

Citation	Method	Description
[6]	Wearable technology for cardiology	Devices of wearable technology were intended for measuring the heart rhythm, heart rate, activity, and thoracic fluid. For classification and understanding, a framework was given to the wearable devices for improving healthcare.

[16]	Technology for cardiovascular disease patient	475 papers from PubMed library were examined for solutions of telemedicine to improve medication adherence of cardiovascular disease patient. 74 articles were assessed. The articles exhibited that suggestions associated with solutions of telemedicine are typically conflictive. The use of SMS was considered for patients regarding their medication because of forgetfulness.

[17]	Big data for monitoring of proactive healthcare of patients of chronic diseases	A system of health proactive monitoring is planned for cardiac patients. In the study, an electronic band is worn by the patient and the real-time situation of health and system of e-health are to process the obtained data from patient. The system supports the patient to take proactive process beside some of the abnormal states in their health and further supports the doctors to monitor the health of patient on a regular basis.
[18]	Deep learning network in left ventricular volumes identification in cardiac MRI	The research has established left ventricular volumes approach of identification without segmentation by deep learning technology and the data set form large-scale cardiac MRI from second annual data science bowl in 2016

[19]	Medical data mining and heart disease	The study offered review of the associated techniques of data mining for finding of diseases classes and heart failure. Additionally, emphasis is given on sequential mining.

[20]	ML horizon in cardiac hybrid imaging	The study presented summary of the fundamental notions in ML and its applications in standard cardiac imaging

[21]	Mobile heart rate monitoring system for patient of MI	Application of mobile for the patient of myocardial infarction (MI) is presented to preserve heart rate tracking and with stress-free pursuing for emergency support

[22]	Clinical guidelines in cardiology run-through in Sudan	Interviews in the two main cardiac hospitals of Sudan were led and an exploratory study among the hospitals' doctors was prepared for examining the perceptions of a huge population of prescribers of the subject examined

[23]	Big health data	Management of cardiac data and operative concept of remodelling to examine early symptoms of heart failure is presented

[24]	Big health data records for early and late translational cardiovascular research	The research censoriously reviewed the challenges of big data before time and after the event stages of research in translational cardiovascular disease

[25]	Factorization of tensor for precision medicine in failure of heart with preserved ejection fraction	The study examined the related woks on factorization of tensor applications in the associated biomedical field of phenotyping and genotyping

[26]	Mobile messaging applications' effect on knowledge of cardiac patients with risk of coronary artery disease and healthy lifestyle adherence	The research led a study from January to April 2017 in Klang Valley's teaching hospital for determining the effect of mobile messaging applications on patients with coronary artery disease and observation of healthy life

[27]	SVM for classification of biomedical signal on IoT platform	The study observed the signal over digital signal processor and then computed the blood oxygen saturation, heart rate, and blood pressure. SVM was considered for the purpose of showing the data and its classification into unhealthy, healthy, and very unhealthy and designates accuracy of classification prediction.

[28]	Heart failure prevention	Risk factors of heart failure and focus on prevention are specified

[29]	Statistical shape models of the heart	The study presented summary of the collected works of statistical shape models in cardiac imaging

[30]	Classifying mining techniques for the accessible clarification for heart disease prediction	Framework to use healthcare data for attributes based heart disease prediction is presented in the study

[31]	Statistical based recommendation model for the patients of heart disease	Smart system of recommendation is presented for patients with heart disease in the fields of medical informatics and e-health

[32]	Modelling 4D for rapid assessment of biventricular function in congenital heart disease	The study has quantified 4D biventricular function from analysis of standard cardiac MRI

[33]	Big database applications and forthcomings in cardiology	Applications of big database studies in cardiology were presented in the study

[34]	Approach of big data to myocyte membrane analysis	The study presented an approach for identification of particular pathological ion dynamics responsible for abnormal electrical behaviour practiced through the experiment

[35]	Distance, quality, or relationship? Interhospital transfer of patients with heart attack	The research inspected the patterns where the patients of heart attack are transferred between the hospitals. The three key factors in transferring destinations are:
		(i) The distance between sending and receiving in hospitals
		(ii) Widely reported quality measures of receiving hospitals as specified by whether they are related with the same multihospital system
		(iii) The relationship between sending and receiving hospitals
[36]	Feature analysis and coronary artery heart disease data sets	Integrate the experimental results of the examination of ML which are applied on varied data sets aiming at the coronary artery heart disease

[37]	Mapping of ventricular tachycardia in patients with heart structural disease	The paper has focused on the procedure of mapping ventricular tachycardia; the conventional and novel technique of mapping and the details of some methodological tips are given

[38]	Patients' baseline characteristics with heart failure and preserved ejection fraction during admission with acute heart failure in Saudi Arabia	Saudi Arabian patients with HFpEF were examined with acute heart failure. The clinical characteristics, signs, and indications of heart failure, echocardiographic findings, and medications during admission and at hospital discharge were determined.

[39]	Cardiovascular dysautonomias diagnosis and treatments through data mining	The authors established a cardiovascular dysautonomias identification system for the prediction of appropriate treatments and diagnosis for patients with cardiovascular dysautonomias through the data set extracted from the ANS unit of University Hospital Avicenne in Morocco

[40]	Approach of data transmission based on adaptive energy efficiency for prediction of heart disease	The research developed an adaptive energy resourceful transmission system which can recognise the important events like myocardial infarction and reduce data transmission from the devices

[41]	Analytics of big data in prediction of heart attack	The study identified the analytics uses in big data for the prevention and prediction of heart attack, privacy of the patients, and the challenges for the use of technology in big data. The study analyzed the national and international databases for the proposed study.

[42]	Cloud computing for myocardial fibre information in vivo	System of cloud-based investigation is intended for cardiac images and link services of computation for remote sharing. A method for postprocessing of image is defined as important service for obtaining information on in vivo myocardial fibres.

[43]	Using big data for assessing the risks of arrhythmia	The research presented an algorithm to involuntarily identify the R, S, and T wave peaks in epicardial electrogram signals

[44]	ML framework and imaging based big data for rapid phenotyping of left ventricular diastolic function	The study proposed that the cardiac biomechanics produce adequate information which can affect ML and framework of big data analytics for function of automated left ventricular diastolic assessment

[45]	Insights from echo reports of paediatric disease of heart	The entity site-feature values are mined in triples in the report of echo and then on the ground of this prediction of the level of risk

[46]	Framework of probabilistic data driven for scoring the preoperatives recipient-donor heart transplant survival	The technique of Bayesian belief networks is used. The approach contains four phases; the first and second phases of the data are preprocessed and a set of predictors are produced based on different variable selection method. The medically associated variables are added to the list of variables in the third phase, and in the last phase the Bayesian belief networks technique is applied.

[47]	Identification of heart arrhythmia through big data-based extraction of fuzzy partition rules	The research presented a novel semiautomatically fuzzy partition rules for facilitating an accurate and robust aspect into cardiac arrhythmia. The approach of text mining is demonstrated and applied to large data set containing freely existing articles in the PubMed library. The information is mined and then put to the experimental data and expert information for facilitating robust system to tackle the issues arising through the assessment of medical big data.

[48]	Big data for prediction of heart disease through map reduction	The research has established a central monitoring system for patients of large set of health records as input. It is intended to mine the essential information from large set of medical records through the method of map reduction. By using this approach, it can be decided whether there is patient normality or abnormality.
[49]	Cardiovascular risk clustering factors highlighted the coronary artery calcium as a strong clinical discriminator	The authors studied the relations between cardiovascular risk clustering and the discriminators of disease of cardiovascular factors

[50]	Mobile health initiatives for cardiovascular disease	The current technological and clinical improvements containing wearable health tracking devices, smartphone devices, and social media for supporting behaviour factors of risk for cardiovascular disease in terms of smoking, physical inactivity, and suboptimal nutrition

[51]	Sudden cardiac death with risk stratification and computational cardiology	The study defined guidelines of what is to be required for making the translational step, through the comparatively well intended cases required or drug induced long QT as a case of syndrome

[52]	Technology of smartphone in cardiology	The research presented various applications of smartphone based technologies in cardiology and gave a review of them

[53]	Visualization of cardiovascular MRI challenges and opportunities	The study offered an overview of the existing associated works of visualization approaches and emphasis on the visualizing imagery issues resulting from 2D myocardial tagging in CMR

[54]	Big data in cardiology	The article's purpose is the three encouraging big data applications in cardiovascular care, with “proof-of-concept” challenges to be met if the encouraging data is to be comprehended

[55]	Cardiovascular medicine big data, health informatics, and future	The study offered a report on cardiovascular medicine big data, health informatics, and future

[56]	Tool for the MIMIC-II database, a web-based data visualization	The objectives of the study are: (a) to build an interactive and (b) data visualization tool based on web MIMIC-II Furthermore, the research mainly offered two features of exploration and comparison. The first feature helps the patient cohort within MIMIC-II and visualized the distribution of various variables including administrative, clinical, and demographic variables within the selected cohort. The second feature helps the users in selection of two patient cohorts and visual comparison with other variables.

[57]	Connecting the dots: from big data to healthy heart	The study designated various sources of big data in cardiology followed by talk over the possibilities of building the best use of data-driven knowledge production models

[58]	Libraries implementation of open-source data visualization of web portal for patients of diabetes	A web portal is employed for improved communications of diabetes patients with doctors for the process of identification and handling of diabetes. Medical data are offered on the portal based on open-source libraries.

[52]	Technology of smartphone in cardiology	The research discusses the details of diverse applications of technologies of smartphone in cardiology

[59]	Machine learning approaches in detection of ischemic heart disease	SVM and Osuna were used for detecting the ischemic disease of heart. The principal component analysis algorithm was also used.

[60]	Paediatric cardiovascular disease in the era of transparency in healthcare using big data	The research offered a review on analytics of big data impact in paediatric cardiovascular disease and its possible issues of transparency in distribution of care

[61]	Data visualization: science on the map	A tool box for data visualization

[62]	Harnessing the heart of big data	The paper discussed the following:
		(i) Report on big data science research
		(ii) Potential of data science to support examinations of cardiovascular diseases
		(iii) Challenges and opportunities

[63]	4D OCT in developmental cardiology	The chapter emphasizes on numerous existing solutions and gives review of the perspective in the evaluation of 4D OCT imaging for cardiovascular system in the past several years
[64]	Kinect-based gesture prediction in volumetric visualization of heart from CMR imaging	The research aims to offer a virtual human heart from medical imaging data with incorporation of collaborating interface using visual 3D holographic, haptic, and sonic feedback

[65]	Feast for the eyes	The research presented the existing data visualization uses and reviewed the probable issues, benefits, and applications of libraries

[66]	Cardiac 4D ultrasound imaging	Overview of the technological developments for volumetric imaging of the heart beat with the support of ultrasound is given

[67]	Probabilistic data-driven framework for scoring the preoperative recipient-donor heart transplant survival	The study presented Bayesian belief network containing four phases. The data is preprocessed in the first two phases and produces a candidate set of predictors. Medical related variables are added in the third phase and, finally, the model of Bayesian belief network is applied.

[68]	Health analytics	The chapter discussed the visualization, analysis, and mining of healthcare data and concludes the way in which data can be proficiently accomplished which further improves the ability of organization to control risk, yield revenue, and cost

[69]	Electrophysiology-morphous merging of human heart based on composite visualization approach	The paper presented cardiac electrical excitation propagation model based on the data of human cardia cross-sectional to discover the cardiac electrical activities. After that, biophysical visualization method is applied for the biophysical integration of cardiac anatomy and electrophysiological properties, which provide the equivalent position, spatial relationship, and the whole process in 3D space with the context of anatomical structure for giving the details of biophysical and electrophysiological activity.

[70]	Big data for cardiology: novel discovery?	The paper determined the encouraging data sets for finding of science and the impact on the approaches used in science in general and explicitly in cardiology

[71]	Visualization of medical volume though intelligent approaches	The uses of algorithms and intelligent approaches of visualizing medical big data are presented. The article discusses the existing software and toolkits for visualization of medical volume.

## Data Availability

No data were used to support this study.
